The article "Decision Scheduling for Cloud Computing Tasks Relying on Solving Large Linear Systems of Equations" was published in 2022. Journal: Comput Intell Neurosci.

# Decision Scheduling for Cloud Computing Tasks Relying on Solving Large Linear Systems of Equations

**DOI:** 10.1155/2022/3411959

**Published:** 2022-03-19

**Authors:** Jing He

**Affiliations:** College of Artificial Intelligence and Big Data, Chongqing Industry Polytechnic College, Chongqing, China

## Abstract

With the continuous reform and innovation of Internet technology and the continuous development and progress of social economy, Big Data cloud computing technology is more and more widely used in people's work and life. Many parallel algorithms play a very important role in solving large linear equations in various applications. To this end, this article aims to propose and summarize a cloud computing task scheduling model that relies on the solution of large linear equations. The method of this paper is to study the technology of solving large-scale linear equations and propose an M-QoS-OCCSM scheduling model. The function of the experimental method is to solve the problem of efficiently executing *N* mutually dependent parallel tasks within limited resources, while fully satisfying users' expectations of task completion time, bandwidth rate, reliability, and cost. In this paper, the application experiment of large-scale linear equations in task scheduling is used to study task scheduling algorithms. The results show that when the task load is 10 and 20, the convergence speed of the MPQGA algorithm is 32 seconds and 95 seconds faster than that of the BGA algorithm, respectively.

## 1. Introduction

The rapid development of the Internet has also promoted the development of cloud computing, and people's research on cloud computing has become more and more in-depth and extensive. Large-scale data mining and distributed processing technology on the Internet have also been paid more and more attention. This paper combines the characteristics of the two and proposes a model combining text mining and task scheduling under cloud computing. Cloud computing is a new business computing model that uses network connections to obtain various applications, data, and IT services. The core of cloud computing is the integrated scheduling and management of cloud environment and task resources submitted by users according to user needs, and users only need to pay on demand. Therefore, for cloud services, how to meet the different needs of different users for quality of service (QoS) is an important issue that needs to be considered when scheduling cloud computing.

The study of resource deployment and task scheduling problems and their solutions in the cloud computing environment is of great significance and value for the theoretical research and application practice of cloud computing. As a business service, cloud computing must not only consider optimizing task scheduling strategies to improve the service capabilities of the system but also consider the service revenue of cloud service providers. There are some controversies in this area, but there is no efficient solution yet. Therefore, studying cloud computing task scheduling strategies has important theoretical value and practical significance for improving the service capabilities of cloud computing systems.

This paper proposes a balanced clone scheduling algorithm that can effectively improve resource utilization and task scheduling efficiency. This paper proposes a model that combines data mining and task scheduling in a cloud environment. Combining the advantages of data mining and distributed computing, this model can calmly deal with data processing of massive amounts of information and provide efficient services for users. This paper comprehensively considers the transmission cost, processing time, processing cost, and transmission time of data in the cloud computing environment, and proposes a mathematical model for task scheduling optimization. And this paper proposes a mathematical model and particle swarm optimization algorithm design based on the increase of the variable neighborhood. The simulation results show that the proposed optimization model and optimization algorithm can not only optimize the time, but also optimize the cost.

## 2. Related Work

The road to solving large-scale linear equations has never stopped. In recent years, people have gradually combined it with task scheduling in order to achieve unexpected results. Wang et al. propose an SSLE method for general constrained optimization based on the mixed exact penalty function. He added automatic adjustment rules to the algorithm for the selection of penalty parameters to ensure that the number of updates of penalty parameters is limited. He also extended the Facchinei activity set recognition technology to general constrained optimization and gave the corresponding recognition function. In each iteration, the algorithm only solves two or three simplified linear equations with the same coefficients to obtain the search direction. Without assuming strict complementarity and weaker than strong second-order sufficient conditions, the convergence rate of the algorithm is proved to be super linear [1]. Phuc and Verbitsky obtained the global solution of quasi-linear equations with metric coefficients and solved a large number of model problems [2]. Lv and Wang studied the existence, uniqueness, and asymptotic stability of traveling wave fronts for discrete quasilinear equations with time delays. He first established the existence of traveling wave fronts using hyperon solutions and monotonic iteration techniques. Then he proved that the traveling wave front is unique before the translation. Finally, he used the comparison principle and compression technique to prove that the traveling wave front has a phase shift and is globally asymptotically stable [3]. Mingtong introduced the basic process of automatic modeling of large buildings. By extending the L-system theory, using elevation maps and automatic river recognition, he researched and proposed an automatic road generation method for complex terrain. Experiments show that the results given by his method are consistent with the surrounding terrain environment. It can automatically generate modifiable roads in complex terrain constrained by altitude and rivers. The road generation algorithm, based on the Voronoi diagram he proposed, can effectively make up for the lack of road changes generated by the system [4]. Samriya et al. proposed a multiobjective penguin optimization algorithm. The proposed method is analyzed through binary gravity search algorithm, ant colony optimization, and particle swarm optimization, which makes it suitable for virtual machines in data centers. Compared with other strategies, the algorithm he proposed is energy-efficient and has significant differences [5]. Jabir et al. proposed an enhanced antlion optimization algorithm mixed with the popular particle swarm optimization algorithm to optimize workflow scheduling specifically for the cloud. The research aims to provide enhanced workflow scheduling that is safer than the existing framework. It enhances the program's ability to evaluate according to cost, load, and completion time [6]. Tang et al. proposed an energy-saving workflow task-scheduling algorithm based on DVFS, whose purpose is to obtain more energy savings and maintain service quality on the premise of meeting deadlines. This algorithm can recycle useful idle time after the server is merged and obtain the entire makespan and deadline based on the heterogeneous-earliest-finish-time algorithm [7]. Gruzlikov et al. proposed a pipeline workshop scheduling method for the calculation process in a distributed real-time system. This method is based on a solvable system with a simple optimization scheduling algorithm. This method opens up ideas for improving the efficiency of the assembly line workshop [8, 9].

## 3. Linear Equations Solution Method and Task Scheduling Method

### 3.1. Common Large-Scale Linear Equation Solving Technology

There are two methods for solving linear equations in direct method and iterative method [10]. Small and medium-sized equations (*n* < 10000) are often solved by the direct method, and the direct method needs to decompose the coefficient matrix A. Under normal circumstances, matrix sparsity cannot be guaranteed. As the degree *n* increases, the amount of memory required becomes O (*n*2), and the amount of floating-point operations required becomes O (*n*3). The sparse direct method based on sorting has some control over memory requirements and time consumption, allowing modern single-CPU personal computers to solve 100,000-order matrices. However, the success of the sparse direct method is related to the nature of the matrix itself, and higher-order linear systems are powerless [11]. Therefore, iterative methods are often used for large or very-large equations. In simple terms, the iterative method is to create a modified *S*_*k*_ for the initial approximate solution vector *X*_o_ of each step. This makes the next approximate solution vector *X*_*k*+1_ equal to the current approximate solution plus the correction vector *S*_*k*_.

(1) $$\begin{array}{c} X_{k+1}=S_{k}+X_{k}. \end{array}$$

This produces an iterative vector sequence {*X*_*k*_}. It can be seen that the ideal correction vector should be

(2) $$\begin{array}{c} S_{k}=X^{*}-X_{k}=Q\left(b-Q\cdot r_{k}\right), \end{array}$$

where *X*^*∗*^ is the solution of the simultaneous equations, and *r*_*k*_ represents the *k*th residual vector. However, in order to obtain this ideal correction vector, this article needs to solve equation *Q·r*_*k*_=*X*_*k*_, which is actually the same problem as solving the original equation. Different iterative methods represent different methods of calculating the correction vector *S*_*k*_ [12]. The classic iterative method is based on matrix division, assuming that the coefficient matrix *A* has the following divisions.

(3) $$\begin{array}{c} A=P-Q, \end{array}$$

where *P* is the invertible matrix and the original system of equations is (*P* − *Q*) *x* = *b*. Therefore, the following iteration sequence is constructed.

(4) $$\begin{array}{c} X=P^{-1}Q_{xk}+P^{-1}b. \end{array}$$

In order to avoid calculating *P*^−1^*Q*_*xk*_ and *P*^−1^*b*, it can turn to solving the equations in the following way:

(5) $$\begin{array}{c} P_{xk}=Q_{xk}+b. \end{array}$$

Different *P* choices have different segmentation methods and different iterative methods [13]. Assumptions:

(6) $$\begin{array}{c} A=D-C_{L}-C_{K}. \end{array}$$

Among them, *D* is the diagonal part of *A*, *C*_*L*_ is the lower triangular part of *A*, and *C*_*K*_ is the upper triangular part of *A*.

In order to achieve better results, people constructed a symmetric over-relaxation method (SSOR method), splitting *A* into *A* = *P*_*ssos*_–*Q*_*ssor*_, where

(7) $$\begin{array}{c} P_{SSOR}=\frac{w}{2-w}\left(\frac{1}{w}D-C_{L}\right)D^{-1}\left(\frac{1}{w}D-C_{K}\right). \end{array}$$

In addition, there are methods such as alternating direction iteration, Hermitian and anti-Hermitian splitting, and multiple splitting, all of which are based on practical problems and are all numerically algebraic [14]. The coefficient matrix of the linear equation system obtained by the finite-element method or the method of moments is generally a complex symmetric matrix, which can be described in the following format.

(8) $$\begin{array}{c} \left(A+iB\right)\left(z+iy\right)=b+ic. \end{array}$$

Among them, *A*, *B* ∈ *R* is a real symmetric matrix. The Krylov subspace method of common asymmetric matrices (such as GMRES, BICGSTAB, and QMR) can be used to solve complex symmetric linear equations. However, using these methods to solve the problem does not take advantage of the symmetry of the matrix. Some solutions transform the symmetric system into an equivalent real symmetric system and then use the Krylov method to solve the real symmetric matrix [15]. The following are some iterative methods for directly solving (8). Using the concept of quasi inner product (*x*, *y*)=*x*^*T*^*y*, where the *x*, *y* ∈ *C* superscript letter *T* represents transpose instead of conjugate transpose, the QMR method can recursively reach the minimum in a short time. This type of quantity and special matrix are often encountered in actual engineering [16]. The key to the success of the Krylov subspace method is the choice of prerequisites. The preprocessing is to transform a linear equation system into another linear equation system with the same solution, but the transformed equation system has the characteristic of facilitating iterative solution. The prerequisite is to generate a matrix for this transformation. If *P* is an invertible matrix somewhat similar to *A*, then the preprocessed system looks like the following equation:

(9) $$\begin{array}{c} P^{-1}A_{x}=P^{-1}b. \end{array}$$

If there is the same solution as equation (1), and there is an equation that is easy to solve, then *P* is called a prerequisite. Equation (9) is preprocessed from the left side and can also be preprocessed from the right side.

(10) $$\begin{array}{c} AP^{-1}y=b,\;x=P^{-1}y. \end{array}$$

Or, preprocess both sides at the same time:

(11) $$\begin{array}{c} P_{1}^{-1}AP_{2}^{-1}y=P_{1}^{-1}b,\;x=P_{2}^{-1}y. \end{array}$$

Then, the precondition in formula (11) is *M* = *M*1M2. A good precondition should have the following two properties: the system after the precondition should be easy to solve, the precondition should be easier to construct and the cost of applying the precondition should not be too high [17].

In modern computer architecture systems, the biggest problem with incomplete decomposition of prerequisites is that it is not easy to parallelize the process of construction and use. Approximate prerequisites for adapting to modern computer structure systems have appeared, and their implementation has natural parallelism [18]. In recent years, the algebraic multigrid (AMG) method that combines the area division (DD) method, multigrid (MG), and physical background to solve partial differential equations (PDEs) has become a hot spot in numerical computing [19].

### 3.2. M-QoS-OCCSM Scheduling Model Based on Cloud Computing

The architecture of the M-QoS-OCCSM collaborative scheduling model proposed in this chapter is shown in Figure 1.

As shown in Figure 1, the execution process of the entire M-QoS-OCCSM scheduling model is as follows. First, the user submits the application task with the deadline of the bottom line and the scheduling budget target constraint to the task scheduler. Then the task scheduler sends the QoS target constraint conditions and other related parameter information of the application task to the extension module of the M-QoS-OCCSM model [20]. Next, the extension module of the M-QoS-OCCSM model first applies the method described in the previous section to model the application task with multiobjective constraints. Then comprehensively consider the application task's QoS target constraints and user expectations and based on a membership function, apply the method described to convert the application task's multiple QoS target constraints into a single-objective constraint optimization problem. Finally, the reconstructed genetic algorithm is applied to approximate the optimal solution of the mentioned single-objective optimization problem [21]. The calculated result is the final scheduling decision plan, which is returned to the scheduler. The scheduler selects appropriate computing resources for the application tasks for scheduling according to the optimization results, thereby completing the scheduling decision.

The extension module serves as an integrated unit in the entire M-QoS-OCCSM scheduling model architecture. For some applications, it can be designed as a separate middleware module for real task-scheduling scenarios [22].

From the user's point of view, the user always hopes to complete all application task scheduling requests within a desired time interval. This means that the actual execution of application tasks should be reduced as much as possible on the assigned computing nodes. At the same time, for a specific resource *R* available on a computing node, the total computing power consumed by all application tasks on the resource *R* cannot exceed the computing power that the resource can provide [23].

It can be seen from the analysis that the QoS target constraint of the aforementioned time limit bottom line can be expressed as follows:

(12) $$\begin{array}{c} \min\left(O_{\text{deadline}}\right)=\overset{T}{\underset{t=1}{\sum }}\overset{N}{\underset{n=1}{\sum }}M_{tn}V_{tn},s.t.\overset{T}{\underset{t=1}{\sum }}\overset{N}{\underset{n=1}{\sum }}\overset{K}{\underset{k=1}{\sum }}M_{tn}R\leq \overset{N}{\underset{n=1}{\sum }}\overset{K}{\underset{k=1}{\sum }}S\left(CN_{tn}\right). \end{array}$$

On the contrary, users always want to save scheduling costs as much as possible while obtaining satisfactory services. Therefore, the cloud system should complete the scheduling and execution of all tasks as much as possible under the constraints of the established scheduling budget [24]. In other words, in an established cloud computing environment, the system should reduce the total scheduling cost of all tasks as much as possible. In addition, for a specific application task *t*, the sum of the scheduling costs consumed by all available resources on the target computing node cannot exceed the task scheduling budget.

According to the analysis, the QoS target constraint of the application task scheduling budget can be expressed as follows:

(13) $$\begin{array}{c} \min\left(O_{\text{budget}}\right)=\overset{T}{\underset{t=1}{\sum }}\overset{N}{\underset{n=1}{\sum }}M_{tn}C_{tn},s.t.\overset{N}{\underset{n=1}{\sum }}M_{tn}C_{tn}\leq B_{n},\forall n\in T. \end{array}$$

This paper compares the algorithm based on QoS constraints with the basic genetic algorithm. The relationship between tasks with interdependence constraints is shown in Figure 2, and the specific parameters and weight vector settings are shown in Table 1.

The user wants to pay as little scheduling cost as possible for the scheduling request of the application task. In real-world cloud computing application scenarios, the cost of scheduling application tasks is often directly proportional to the user's satisfaction with completing the scheduling goals. Therefore, users want to spend less on their application task scheduling budget, assuming they have a satisfactory scheduling service [25]. As shown in formula (14), assuming that a satisfactory scheduling service is obtained, the membership function of the task scheduling expenditure can be used to express the membership of the task scheduling budget and the scheduling target.

(14) $$\begin{array}{c} Y_{\text{nm}}^{\text{budget}}=1-\frac{C_{\min}}{C_{nm}}. \end{array}$$

In the formula, *C*_min_ represents the minimum expected value of the scheduling overhead of the application task *t*_*n*_, and *C*_*nm*_ represents the scheduling budget when the application task *t*_*n*_ is scheduled on the target computing node *C*_*nm*_. It can be seen from equation (14) that as the scheduling budget expenditure *C*_*nm*_ of the application task *t*_*n*_ decreases, the membership function value *Y*_*nm*_^*bu*  *dg*  *et*^ of the scheduling budget decreases. Since users want to pay as little task scheduling budget as possible, the goal of the final task scheduling solution is to minimize the value of the mentioned membership function as much as possible [26].

Through the analysis of the two QoS target constraints, deadline and scheduling budget. This article finds that with less scheduling budget and the shortest possible deadline, everything needed to complete an application task scheduling request has increased. It tries to minimize the aforementioned period. The membership function value of time and the membership function value of scheduling budget expenditure. Based on this conclusion, two membership functions can be used to transform the task scheduling multi-QoS objective constraint optimization problem into a single-objective constraint optimization problem. The transformed single-objective constrained optimization problem is shown as follows:

(15) $$\begin{array}{c} \min\left(O\right)=w_{1}\min\left(O_{\text{deadline}}\right)+w_{2}\min\left(O_{\text{budget}}\right). \end{array}$$

In the formula, the deadline and scheduling budget weight parameters *w*_1_ and *w*_2_ satisfy ∑_*n*=1_^2^*w*_1_=1, 0 ≤ *w*_1_ ≤ 1. When scheduling tasks, pay attention to the deadlines and the scheduling budget constraints of each user. Therefore, when constructing the objectives of the mentioned task scheduling scheme, adjusting the two weight parameters for different users can meet the various QoS target constraints of users.

By default, Hadoop usually adopts a first-come first-serve strategy. The advantages of this strategy are simplicity and low overhead, while reducing the burden of the job tracker [27]. The basic idea of solving the problem is to queue up all tasks submitted by the end customer according to the time when the job was submitted. The execution order of the job queue is usually determined by priority and transmission order. That is, the job submitted first by the system has a higher priority by default and will be processed earlier. But the disadvantage of the FIFO strategy is that it is unfair. According to the solution idea of this strategy, for those jobs with low priority, the chance of being processed will be greatly reduced, and the waiting time for idle machines will be particularly long. That is to say, it is difficult to guarantee the QoS for jobs with low priority. This strategy lacks consideration of differences in job requirements.

### 3.3. Cloud Computing Task Scheduling Strategy

Cloud computing resources include storage resources, computing resources, network resources, and so on. In fact, these resources are abstracted into services through virtualization technology and provided to the outside world. On the contrary, there is a correlation between service quality and resource occupancy rate, service quality, and energy consumption. Therefore, when optimizing resources, this article must consider comprehensively, rather than biasing one aspect. Therefore, when optimizing resource deployment and scheduling, all resources must be fully considered and jointly managed and optimized. It is necessary to optimize the QoS, while optimizing energy consumption and cost [28].

The state of task scheduling in the cloud computing environment can be explained as follows. The total number of resources is *P*, and the corresponding set is *R*={*r*1, *r*2 ⋯ *rn*}. The total number of jobs submitted by users is *M*, corresponding to set *J*={*J*1, *J*2 ⋯ *JM*}. Assuming that the *M* jobs corresponding to the set *T*={*T*1, *T*2 ⋯ *TN*} are divided into *N* tasks, the *Jm*th job is divided into *T*_*Num*_(*Jm*) tasks, and then the total number of tasks corresponding to the total number of tasks is as follows:

(16) $$\begin{array}{c} N=T_{\text{total}}\left(M\right)=\overset{M}{\underset{m=1}{\sum }}T_{\text{Num}}\left(Jm\right). \end{array}$$

Network bandwidth is an important indicator to measure network usage [29]. The size of the bandwidth determines the size of the network transmission capacity, which in turn affects the communication efficiency in the cloud environment. The more frequent the communication, the greater the amount of information, and the higher the bandwidth requirements. Let *B*_*wn*_ be the resource bandwidth of the cloud computing environment, *B*_user_ represents the expected bandwidth of the job *Jm* specified by the user, and *B*_*i*_ represents the expected bandwidth of the task *T*_*i*_ divided by the job *Jm*, then

(17) $$\begin{array}{c} B_{\text{user}}=\overset{T_{Num}\left(Jm\right)}{\underset{m=1}{\sum }}B_{i}. \end{array}$$

The function of user satisfaction *w* obtained bandwidth is as follows:

(18) $$\begin{array}{c} W=\left[\frac{\theta }{T_{Num}\left(Jm\right)}\right]\overset{T_{\text{total}}\left(M\right)}{\underset{m=T_{\text{total}}\left(M-1\right)}{\sum }}\ln\left(\frac{B_{wn}}{B_{i}}\right). \end{array}$$

Assuming that the resource failure rate in the cloud computing environment is *P* (which can be obtained through the resource monitoring system) and the user's expected task completion rate is *P*_*succ*_, the user satisfaction function of the job completion rate is as follows:

(19) $$\begin{array}{c} W_{succ}\left(Jm\right)=\theta \;\ln\left[\frac{\left(1-p\right)}{P_{\text{succ}}}\right]. \end{array}$$

Cost constraint is one of the most popular QoS constraints, and cost is one of the important components of user QoS. Assuming that resources are billed per unit, *P*_*i*_ is the number of resources, and *C*_*cpu*_, *C*_*men*_, *C*_*stor*_, and *C*_*BW*_ represent the prices of CPU, memory, storage, and bandwidth resources. Then, the total cost of task *T*_*i*_ can be expressed as follows:

(20) $$\begin{array}{c} C_{i}=P_{1}C_{cpu}+P_{2}C_{\text{men}}+P_{3}C_{stor}+P_{4}C_{BW}. \end{array}$$

Through the previous related research on the existing results of the equations solution, it can be found that each equation solution must have a suitable data center network structure, such as a centralized structure, a distributed structure, and a hierarchical structure [30]. In view of this, before introducing the DRMS equation solution introduced by the task scheduling system architecture in the cloud computing environment, first introduce the data center network structure that implements the equation solution.

As shown in Figure 3, the data center that implements the DRMS equations solution is a hierarchical structure. This structure is mainly composed of three types of nodes: regional host node, regional head node, and ordinary host node (also called site, or Site) [31].

## 4. Task Scheduling Experiment and Analysis Based on Cloud Computing

### 4.1. Application of Large-Scale Linear Equations in Task Scheduling

In mathematics, the Gaussian elimination method is also known as the Gauss Jordan elimination method, which is an algorithm for solving linear algebra system problems using linear equations [32]. The algorithm first determines the rank of the matrix, and then calculates the inverse of the invertible square matrix. When designing the Gauss method that can cancel the inverse allocation process, the elimination method also reduces the unknown coefficients on the main diagonal to zero. The elimination method does not need to replace the diagonal coefficient matrix equation, this method is called Jordan elimination method. However, the number of multiplication and division operations in Jordan elimination is twice that of pure Gaussian elimination. This is not desirable when solving linear equations, but it is useful when solving inverse matrices.

The operating speeds of Gauss elimination method, and Jordan elimination method are shown in Tables 2 and 3, respectively.

The experimental results are shown in Table 4 by running the Gauss elimination method on a 4-core multiprocessor to process the Poisson equation. From the data in the table, the speedup for solving the Poisson equation under four cores can be calculated as shown in Figure 5.

The following conclusions can be drawn from analyzing the graphs in this article: ① When the scale of meshing reaches a certain level, compared with the serial solution of single-core, the parallel solution of four-core will highlight its advantage in solution time. Because, when the scale of grid division is small, the communication time between each process takes a larger proportion than the overall running time. Therefore, the parallelism of multiple cores does not show its advantages in the process of solving a smaller meshing scale. ② Analyzing the speedup ratio of various improved parallel algorithms in Figure 5, it can be seen that the nonblocking method can indeed improve the efficiency of parallel solving. And on this basis, overlapping a part of the calculation with nonblocking message passing can further improve the efficiency of parallel solving. ③ From the analysis of the speedup ratio of the parallel algorithm in Figure 5, it can be seen that if the number of processes is fixed, the parallel efficiency will increase as the size of the subdomain problem increases. As the problem grows, the number of Gauss–Jordan iterations also increases. Moreover, the increase in the number of iterations of the Gauss elimination method has a linear trend with the increase of the grid division scale, which shows the rationality of solving large-scale sparse linear equations by the Gauss elimination method. This paper also proposes a task scheduling optimization strategy based on service quality optimization, taking into account system load conditions. This article also gives the approximate service cost of the system and its related proofs. Through experiments, this article analyzes the model and TSSQO strategy in detail and compares them with representative strategies. It verifies that the strategy in this article can more reasonably schedule tasks, so that the entire system can not only achieve high service quality, but also relatively low service costs.

### 4.2. Multimode Automata Matching Experiment

Most application services in cloud computing must be decomposed into several subtasks for scheduling, and the decomposed subtasks have different degrees of dependence. How to improve the parallelism, real-time and dynamics of coupling-dependent task scheduling, improve system utilization, and perform reasonable scheduling, and deployment of dependent task requests has become a hot spot to be solved in current distributed computing and cloud computing.

This experiment tests the time performance of the multimode automata matching method. The tested hardware environment is 200G hard disk, 16G memory, and two 4-core CPUs. The computer operating system is Ubuntu Linux. This experiment tested the matching algorithm on a 1G data set file and compared the time consumption of the traditional algorithm and the multimode automata algorithm when the comparison rules are the same.

It compares the scheduling length and communication overhead performance of TDDPS with HEFT and Min_Min algorithms in a distributed system composed of three heterogeneous processor nodes with different task sets. And its statistics use TDDPS algorithm to carry on the system load balance that depends on the task scheduling.

The task graph is randomly generated in the experiment. The number of nodes in each task graph [1∼100], task dependencies, the amount of communication data between nodes [1∼100], and the execution time of each task on different processors [1∼100] are all randomly generated. The experiment compares the three scheduling ideas from the three aspects of scheduling length, communication energy consumption, and node resource utilization.  Figure 6 shows the scheduling length and communication overhead of the three on different task sets.

According to the results of Figure 6, it can be seen that the TDDPS algorithm has good performance in terms of scheduling length and communication overhead. Owing to the distributed negotiation and scheduling mechanism, each execution node in the heterogeneous system first evaluates the load of the node, and it makes a negotiation response message to the task request according to the real-time load situation of the node. This ensures a certain degree of load balance and improves resource utilization.

In order to test the performance of the BCSOA algorithm, this paper uses the CloudSim simulation platform to simulate and build a data center. At the same time, the algorithm is compared and tested with the DFGA algorithm and the ASAP algorithm. At present, the ASAP algorithm and the DFGA algorithm are typical algorithms in the field of cloud computing task scheduling research. It has achieved relatively ideal experimental results in the specific application process.

The experimental test contains two aspects: the first type of experiment is mainly compared from the perspective of task completion time, and the second type of experiment is mainly compared from the perspective of the balance factor.  Figure 7 shows the comparison of the task completion time of the three task scheduling algorithms when the number of tasks in the system is *n* = 1000.

Experimental data show that the traditional matching algorithm has severe time performance degradation when the number of rules increases, and the matching mechanism using multimode automata can greatly improve the matching speed when the rule set is large. Through the comparison of the results of the four rule sets, the time performance of the matching based on the multimodal automata has been greatly improved compared with the traditional algorithm.

### 4.3. Task-Scheduling Algorithm

In order to verify the performance of the MPQGA task-scheduling algorithm, this paper compares the algorithm with the previously mentioned heuristic algorithms HEFT-T, HEFT-B, CPOP, and the basic random search algorithm BGA. This article carried out related tests on two test sets of actual application program graph and randomly generated DAG application table.

The MPQGA algorithm is implemented by C programming. The DAG task graph is represented by a class, and its members include a series of tasks. It uses a two-dimensional matrix to represent the computing speed of each task in a heterogeneous processor and uses another two-dimensional matrix to represent the amount of communication data between each pair of tasks. The task in the program is also a class, and its members include the predecessor and successor of the task, the input and output of the task, and the amount of data calculation of the task. To implement an FFT with an input vector of *k*, there are 2*k *− 1 recursive calls and *k* log2*k* butterfly operations (this article assumes that *k* = 2*i*, *i* is an integer). In the FFT task graph, each path from the start of the task to the end of the task is a critical path. As the computational cost of tasks at any level is the same, the communication costs of all paths between the two levels are the same.  Figure 8(a) shows the average SLR of the task scheduling algorithm for FFT task graphs of different sizes, in which the MPQGA algorithm is better than the average SLR of other algorithms.  Figure 8(b) shows the efficiency of different algorithms with 64 data nodes, and the MPQGA algorithm is also better than other algorithms in efficiency.

In the experiment of this article, the value of CCR is set to 0.2, 0.4, 0.6, 1.0, 5.0, and 8.0.  Figure 9 shows the average SLR and the efficiency value of the algorithm with different CCR values and different numbers of heterogeneous processors.

Figure 9(a) shows that when the CCR value increases, the average SLR of the algorithm also increases.  Figure 9(b) shows the efficiency of the algorithm in the case of different numbers of processors.

In these experiments, this paper uses randomly generated task graphs to evaluate the performance of the algorithm. In order to generate random graphs, this article implements a random graph generator that allows users to generate random graphs with different characteristics. The input parameters of the generator: the number of tasks in the graph, the number of instructions for each task (calculation), the number of subsequent tasks (parallelism), and the CCR value. This article evaluates the performance of the algorithm under different parameters, including different numbers of tasks, different numbers of heterogeneous processors, and different CCR values. The value in Figure 10 is the average maximum and minimum completion time of more than 100 different random DAG graphs.

Figure 10 shows the convergence process of the maximum completion time for a set of randomly generated DAG application graphs (size 10 and 20, respectively). This article can observe that when the DAG application graph is small, the convergence speed of the MPQGA algorithm and the BGA algorithm is very fast. When the DAG application becomes very large, the convergence speed of the algorithm becomes slow, but the convergence speed of the two algorithms is different. The MPQGA algorithm proposed in this paper converges faster than the BGA algorithm, and the final minimum and maximum completion time obtained is better than the BGA algorithm.

In general, with the development of network reliability, cheap computer hardware and software, virtualized hardware technology, and service-oriented architecture, more and more companies have begun to invest in the development and application of cloud computing technology. More and more companies and individuals are beginning to use cloud computing technology. It continues to promote the progress and development of cloud computing technology. Today, cloud computing, as the core of the next generation of IT technology, has great advantages such as high flexibility, scalability, ease of use, economies of scale, green energy saving, and environmental protection. It is considered to be the next-generation network after the Internet.

## 5. Discussion

Cloud computing has become a trend in the field of IT technology. This article has conducted in-depth research on the task scheduling strategy of cloud computing and has achieved some results. Nevertheless, the work of this article is not yet full and mature enough. At the same time, due to the rapid development of cloud computing technology, there are still many problems in the field of cloud computing technology that need to be further improved and resolved. These problems are mainly reflected in the following aspects: user privacy and data security. The development of cloud computing requires the participation of a large number of users. How to ensure that the user information stored in the cloud is sufficiently safe to ensure that user privacy and user data will not be collected or leaked by cloud service providers and will not be stolen or illegally used by third parties. This is not only a technical issue but also a legal issue. It needs the joint promotion of researchers and government departments. Scholars in the future should strengthen the study of compressed storage of sparse matrices. In this article, the matrix storage of the MPI experiment program is a file that stores all zero elements in the sparse matrix, which will greatly waste the system's memory resources and affect the performance of the parallel program.

## 6. Conclusion

This paper has conducted in-depth analysis and research on the task-dependent scheduling mechanism in cloud computing, including the characteristics and shortcomings of the existing scheduling model, and the problems to be solved by task-dependent scheduling. This paper proposes a new system model suitable for cloud computing environment and a dynamic parallel dependent task scheduling mechanism. In this paper, aiming at the resource-matching problem in the scheduling process, a parallel matching method based on multimode automata is proposed. When the task amount is 10, the calculation speeds of the BGA algorithm and the MPQGA algorithm are 43 and 11, respectively, and when the task amount is 20, the calculation speeds of the BGA algorithm and the MPQGA algorithm are 108 and 13, respectively. It can be seen that the MPQGA algorithm is more excellent, and the more tasks, the more obvious the advantage.

## Figures and Tables

**Figure 1:** M-QoS-OCCSM system architecture.

**Figure 2:** Interdependence diagram between tasks.

**Figure 3:** Cloud computing data center network structure diagram.

**Figure 4:** Speedup analysis of two elimination methods (two nodes).

**Figure 5:** Speedup ratio of Poisson equation solution under quad-core.

**Figure 6:** Comparison of scheduling length and communication energy consumption of different task sets on three nodes.

**Figure 7:** Comparison of task completion time of three task scheduling algorithms (*n* = 1000).

**Figure 8:** Algorithm average SLR and efficiency of fast Fourier transform: (a) algorithm average SLR vs. FFT graph size and (b) algorithm efficiency vs. number of processors.

**Figure 9:** Algorithm average SLR and efficiency of molecular dynamics code: (a) algorithm average SLR vs. CCR and (b) algorithm efficiency vs. number of processors.

**Figure 10:** The convergence speed of the algorithm under different number of tasks: (a) number of random tasks = 10 and (b) number of random tasks = 20.

**Table 1:** Task scheduling algorithm parameter setting table.

	Two task scheduling algorithms
Total resources	15
Total number of tasks	45
Unit price of virtual machine resources	7
Virtual machine computing performance (million instructions per second)	1500
Task length (one hundred instructions)	10,000
Virtual machine resource bandwidth (Mb)	1024
Expected time (seconds)	65
Expected bandwidth (Mb)	910
Expected cost	4500
Number of generations	125
Crossover probability parameter	*k*1 = 0.6, *k*2 = 0.8
Mutation probability parameter	*k*3 = 0.2, *k*4 = 0.06
Variation gene range parameter, *d*	5

**Table 2:** Experimental data of Gauss elimination method.

Number of parallel nodes	Dense matrix scale	1002	2002	5002	6002	9002
	Total time	0.053	0.0817	0.0093	0.1104	0.0523
	Communication time	0.0576	0.0994	0.0935	0.099	0.0254
1	Parallel computing time	0.0446	0.0064	0.0344	0.1106	0.0059
	Speedup ratio	—	—	—	—	—
	Parallel efficiency	—	—	—	—	—
	Total time	0.1128	0.0884	0.0534	0.0554	0.0488
	Communication time	0.0777	0.0155	0.0955	0.1121	0.0932
2	Parallel computing time	0.0574	0.0069	0.0928	0.1062	0.0052
	Speedup ratio	0.67	0.53	0.31	0.85	0.85
	Parallel efficiency	0.33	0.92	0.99	0.39	0.49
	Total time	0.1069	0.0932	0.0617	0.0501	0.0181
	Communication time	0.0988	0.0045	0.0873	0.0056	0.044
4	Parallel computing time	0.0101	0.0868	0.0439	0.0328	0.0838
	Speedup ratio	1.12	0.9	0.88	0.98	0.68
	Parallel efficiency	0.4	1.19	0.51	0.3	0.64

**Table 3:** Experimental data of Jordan elimination method.

Number of parallel nodes	Dense matrix scale	2002	4002	5002	6002	10002
	Total time	0.0443	0.1012	0.0583	0.0034	0.1169
	Communication time	0.0676	0.0461	0.1171	0.0917	0.0782
0	Parallel computing time	0.006	0.1163	0.1053	0.0995	0.04
	Speedup ratio	—	—	—	—	—
	Parallel efficiency	—	—	—	—	—
	Total time	0.0699	0.0479	0.0687	0.0279	0.0364
	Communication time	0.048	0.0936	0.0636	0.0055	0.0449
3	Parallel computing time	0.099	0.0802	0.0514	0.1047	0.1189
	Speedup ratio	0.39	0.43	0.57	0.45	0.4
	Parallel efficiency	0.55	0.77	0.38	0.61	0.45
	Total time	0.0935	0.0582	0.1137	0.0265	0.063
	Communication time	0.0772	0.0392	0.0976	0.0854	0.0878
4	Parallel computing time	0.119	0.0998	0.033	0.1005	0.0662
	Speedup ratio	0.48	0.62	0.97	0.83	0.7
	Parallel efficiency	0.43	0.63	0.49	0.68	0.73

The comparison of parallel efficiency in various situations is shown in Figure 4.

**Table 4:** Poisson equation solving experimental results (unit: second).

Type of equation	30 × 60	60 × 120	90 × 180
Single core nonimproved	0.228	2.396	11.643
Quad-core nonimproved	0.510	2.240	11.648
Quad-core improvement (nonblocking)	0.479	2.442	11.133
Quad-core improvement (overlapping communication)	0.519	2.284	9.620
Gauss elimination method selection times	0.325	2.595	11.882

## Data Availability

The data used to support the findings of this study are available from the corresponding author upon request.
